# Translation and Expression of Professional Terms of Public Emergencies in External Reports

This article has been retracted.

**DOI:** 10.1155/2022/8973525

**Published:** 2022-09-30

**Authors:** Zhanwei Zhu, Chenhui Wang

**Affiliations:** School of Foreign Languages, Hubei University of Automotive Technology, Shiyan, 442002 Hubei, China

## Abstract

In order to better grasp the expression and translation methods of professional terms in the process of external reporting of public emergencies and grasp the characteristics and elements of the translation of publicity events, this study takes public emergencies as the research object and focuses on the application of English and Chinese professional terms and translation strategies in the process of external reporting. Therefore, based on the in-depth analysis of the news reporting framework of public health emergencies, this paper deeply summarizes the application skills of professional terms in publicity texts, so as to provide a certain reference for further improving the translator's ability to control the means of discourse cohesion and the level of discourse control of Chinese-English professional terms in the translation of public health events.

## 1. Introduction

Foreign news reports are more oriented to foreign and international news media to publicize domestic news content, so from the perspective of publicity, foreign news reports belong to “information language items.” The main function of this kind of discourse is to spread information and provide new knowledge, report the domestic and foreign policies and all aspects of the country to foreign media and foreign audiences, and provide all kinds of information about the country, including economic development information and public event information. However, due to the particularity of public emergencies, we should grasp the expression of professional terms when carrying out external publicity and reporting, so as to avoid the distortion of news information. Therefore, we should not only express the information of public emergencies concisely but also reflect the accuracy of word meaning. This paper is based on this, to explore the translation and expression strategies of public emergencies in the publicity text in depth.  Figure 1 shows the process of translating manuscripts by translation companies [1].

## 2. Literature Review

Bylina et al. pointed out that translation is essentially an act of information transformation and dissemination. Generally speaking, translation is to change one language into another while keeping the connotation of information unchanged. In the process of translation, the translator needs to have a deep understanding of the original text and be able to grasp the text as a whole from the aspects of content, style, and coherence. If you want the translation to be coherent, you have to do a good job of cohesion. Cohesion is one of the important means to achieve coherence. If there is a problem with cohesion, the small will affect the fluency of the article, and the large will change the meaning of the text [2].

Shen believes that publicity translation is to translate many information related to China from Chinese into non-Chinese and then spread by books, newspapers, periodicals, radio, television, Internet, and other media. Publicity translation covers many aspects including politics, economy, culture, and military. Its purpose is to objectively and truly introduce Chinese culture, national conditions, etc. At the same time, it also meets the needs of communication and is easy for foreign readers to accept [3].

Xie et al. put forward two concepts of semantic translation and communicative translation. Semantic translation maximizes the contextual meaning of the original text on the premise of the semantic structure and syntactic structure of the target language. Communicative translation is to make the target language readers and the source language readers get the same information reception effect as much as possible. Due to the different functions and audiences of each text, the focus of these two translation strategies is also different. Take publicity texts for example. When translating, we should not only reasonably adopt the strategy of semantic translation to accurately convey the factual information in the original text but also adopt the strategy of communicative translation as appropriate to make the translation easy to be accepted by foreign audiences and achieve good publicity effect [4].

Chen and Cui pointed out that the most prominent feature of publicity texts is the use of a large number of cohesive devices. The rational use of cohesive devices can make the translation more coherent, and coherence is one of the important conditions for accurately conveying the information of the translation. The commonly used cohesive devices in publicity texts include reference, substitution, ellipsis, connection, and lexical means. Due to the formality of style, publicity texts have a high standard for the logic and coherence of language, and cohesive devices are one of the important means to achieve this standard [5].

Ramesmayer et al. pointed out that cohesion is a semantic concept, which refers to the meaning relationship of idioms. If we want to understand the meaning of a component in a text, we need to refer to another component, and the cohesion relationship will arise. It also points out that there are two types of textual cohesion means, namely, grammatical means and lexical means, and textual cohesion includes intrasentence cohesion and intersentence cohesion [6].

## 3. Analysis on the External Reporting Framework of Public Health Emergencies

Take the “poison capsule incident” as an example. On April 15, 2020, it was exposed that gelatin manufacturers in cities A and B used industrial gelatin with excessive chromium to manufacture capsules [7]. Among them, 13 batches of capsule drugs from 9 pharmaceutical factories represented by the correction pharmaceutical industry contain excessive metal chromium, which is found by relevant departments to be the most serious exceeding times the national standard. The “poison capsule incident” has become a hot topic of public discussion, causing widespread public concern about drug safety.

### 3.1. Sample Survey of News External Reports

This study takes a total of 20 days from April 15, 2020, to May 4, 2020, as the research period. During this period, CCTV news channel's “weekly quality report” column broadcast the special investigation news “secrets in the capsule” to expose the event for the first time, which was reprinted and tracked by many domestic news websites. The “poison capsule incident” instantly became a hot spot of media focus [8, 9]. Within 30 days after the “poison capsule incident” was exposed on April 15, 2020, the number of news reports on the “poison capsule incident” by major domestic media was about 107790 (including reprinted news). According to the number, they are as follows: online media (99585), newspaper media (6720), forum articles (894), and TV media (591).

According to the public opinion monitoring of the “toxic capsule incident” report (as shown in Figure 2), after the “toxic capsule incident” broke out on the 15th, the number of major media reports rose sharply and peaked the next day, and the number of reports on the 17th to 20th showed a downward trend but still remained at a relatively high level and began to fall back on the 21st. On the 23rd, a canal in city A was filled with empty capsules, which attracted attention. The amount of information rebounded, and there was a small upsurge in reporting. From the 24th to the 28th, the amount of events reported gradually fell and tended to be stable. From May 29 to May 4, the amount of media coverage of the event has been hovering at a low level, indicating that the attention of public opinion has declined. After May 4, the amount of news coverage showed a downward trend. The event entered a dormant period of public opinion, gradually faded out of the sight of the media, and temporarily ended [10].

### 3.2. Category Construction

According to the needs of research, this study designed the following categories: report layout, report genre, report theme, source of information, report protagonist, and report position, as shown in Table 1 [11, 12].

Report page is mainly for the category set up by the sample extraction of the newspaper media “Southern Metropolis Daily,” which is mainly divided into front page, important news page, comment page, domestic page, international page, economic page, local news page, and urban page.

### 3.3. Content Analysis of News Reports

As shown in Table 2, the data analysis of report layout is mainly aimed at the categories set up by the newspaper media Southern Metropolis Daily. Layout refers to the arrangement and layout of news manuscripts in the newspaper, which makes readers' first impression of news reports. Layout language is an important way for newspapers to guide public opinion [13]. Note the following: as the cover of the newspaper, the front page of “Southern Metropolis Daily” generally plays the role of reading guide. The specific content is in other pages, so the data on the front page will not be specifically analyzed.

From Figure 3, we find that the distribution of the number of news reports on the “poison capsule incident” in the page of Southern Metropolis Daily is mainly concentrated in the important news section, local news section, comment section, and economic section, of which the important news section (40.9 yuan) accounts for the largest number of reports, highlighting the importance that Southern Metropolis Daily attaches to the “poison capsule incident,” and the important news section is used as “a means of newspaper speech.” In the process of information transmission, readers' attention to this event has been improved [14, 15]. Secondly, the local news edition (19%) mainly includes the news reports of the Pearl River Delta covered by the Southern Metropolis Daily. The local news edition also accounts for a large proportion of the “poison capsule incident,” reflecting the regional characteristics of the news reports of the Southern Metropolis Daily. The comment page (15.1%) mainly includes the editorial part of Southern Metropolis Daily, which is relatively open to express the position of Southern Metropolis Daily on the “poison capsule incident.” The economic edition (10%) mainly includes relevant reports on the impact of the “poison capsule incident” on the economic field. The number of reports in this edition is also large, which is related to the distribution area and audience of Southern Metropolis Daily. Southern Metropolis Daily is mainly sold in economically developed regions such as the Pearl River Delta, Hong Kong, and Macao. Among its readers, social elites and white-collar readers account for a high proportion. Therefore, Southern Metropolis Daily has a broader perspective on the “poison capsule incident.”

From Table 3 and Figure 4, it can be seen that the reporting styles of “poison capsule incident” in Southern Metropolis Daily mainly include news (56.3%), comments (18%), communications (15.2%), and popular science abstracts (6%), of which the news accounts for the largest proportion [16]. At the same time, Southern Metropolis Daily also has a large amount of comments on “poison capsule incident,” which is in line with the style that Southern Metropolis Daily regards current commentary as Qixia.

Figure 5 and Table 4 show the theme distribution of “poison capsule incident” reported by Southern Metropolis Daily. It can be seen from the figure that the news theme of “Southern Metropolis Daily” is “quality inspection and problem capsule treatment” (including off shelf, shutdown, return, and destruction), accounting for the largest proportion of 30.3%, followed by “incident investigation,” accounting for 24%, the “government measures and disposal of relevant responsible persons” accounting for 23%, the “others” accounting for 16.7%, the “star endorsement” accounting for 4.5%, and the case report accounting for 1.5% [17]. The topics with a large number of news are “quality inspection and problem capsule treatment,” “event investigation,” and “government measures and disposal of relevant responsible persons,” and there is insufficient attention to “case report” and other topics.

It can be seen from Figure 6 and Table 5 that the sources of information reported by Southern Metropolis Daily on the “poison capsule incident” are relatively diverse, but the main source of information is government departments and government officials, accounting for 48.5%, followed by media reporters, accounting for 28.8%, experts and scholars, accounting for 10.6%, enterprises and principals, accounting for 6%, and others, accounting for 4.6%, while the proportion of relatively disadvantaged consumers in the “poison capsule incident” is only 1.5%. It can be seen that government officials are easier to access and use media than consumers [18, 19].

It can be seen from Table 6 and Figure 7 that the protagonists of the “poison capsule incident” report of Southern Metropolis Daily are mainly “government departments and officials,” accounting for 33.3%, followed by “industrial and commercial enterprises and principals,” accounting for 32%, followed by drug safety knowledge, accounting for 13.6%, and policies and regulations, accounting for 7.6%. In addition, consumers and stars account for 3%, respectively, and other protagonists account for 6%. It can be seen that in the report of the “poison capsule incident,” Southern Metropolis Daily paid more attention to “government departments and officials” and “enterprises and principals.”

It can be seen from Table 7 and Figure 8 that the reporting position of Southern Metropolis Daily on the “poison capsule incident” is mainly neutral and objective, accounting for 74.2%, followed by negative, accounting for 18.2%, and finally positive, accounting for 7.6%. The proportion of negative reports is greater than that of positive reports, which reflects the outspoken characteristics of Southern Metropolis Daily and plays a positive role in public opinion supervision.

## 4. External Reporting Strategies of WeChat Official Account and Other Media

### 4.1. The Amount of Reports Fluctuated Greatly, and the Outbreak Period Reached Its Peak

The number of COVID-19 reports on the government official account “healthy China” ranks second among the three categories of official account, with 1804, roughly half of the “surging news” on the media official account. From the four stages of the epidemic development, the amount of reports of “healthy China” fluctuated greatly in each stage [20]. On March 9, 2020, Jianghan Fangcang Hospital, the largest Fangcang hospital in B, announced its closure, and the COVID-19 entered a continuous period. In the middle and late March, the number of new infections in many parts of the country fell to 0, and the epidemic was controlled as a whole. The number of reports of “healthy China” contracted to about half of the outbreak period, to 435. On April 8, 2020, B was “unsealed,” and the epidemic development came to the recovery period. Obvious progress was made in the resumption of work and production and classes in various regions, and various industries began to return to normal operation. However, at the same time, in order to prevent the rebound of the epidemic caused by a large number of population movements, the relevant epidemic prevention measures are still not lax, such as the implementation of the serving of individual dishes and the control of the flow of people in public places of entertainment. Compared with the duration, the number of reports at this stage fluctuated slightly, rising slightly to 532. The details of reports in different periods are shown in Figure 9.

### 4.2. Evening Reports Are the Main Ones, While Morning and Afternoon Reports Have Increased Significantly

On the whole, since the gestation period, “healthy China” has remained dominated by evening reports, but the number of reports has increased significantly in the morning and afternoon. On the one hand, it is conducive to releasing relevant important information in a more timely and rapid manner, such as refuting rumors of false information and the route and whereabouts of infected people. On the other hand, due to the strict home isolation measures implemented throughout the country during the epidemic, the traditional work and rest time has changed, and the audience has relatively sufficient time to browse information in the morning and afternoon but also has greater demand for important information. The specific situation is shown in Figure 10 [21].

In terms of the distribution of push time, the push time of “healthy China” in each stage is mainly 19:00-24:00 in the evening, accounting for or close to half of the total. At the same time, through the analysis of samples, it is also found that the number of reports of “healthy China” in the morning between 8:00 and 10:00 in the brewing period is zero, while in the outbreak period, duration period, and recovery period, the number of reports in this period increased to 82, 37, and 88, accounting for 10.3%, 8.5%, and 16.5%, respectively, which is significantly higher than that in the brewing period [22]. In addition, in the afternoon between 13:00 and 17:00, the proportion of reports of “healthy China” in the outbreak period, duration period, and recovery period also increased significantly compared with the gestation period. Accordingly, the proportion of reports from 17:00 to 19:00 decreased compared with the gestation period.

### 4.3. Pure Text and Graphic Forms Are Mainly Used, While Video Reports Have Increased

In terms of content presentation, “healthy China” is mainly in the form of pure text and graphics in all stages, but there are also differences in each stage. The main performance is that in the outbreak period and duration period, the proportion of reported content in the form of video increased significantly compared with the brewing period, and the proportion of video reports in the outbreak period was the highest in the four stages, reaching 35%, and fell back to the level roughly equal to the brewing period in the recovery period, as shown in Figure 11 [23].

### 4.4. Short Stories Dominated, and Medium and Long Ones Increased

As shown in Figure 12, in terms of the length of the report, “healthy China” is mainly 0-5000 words in each stage, accounting for nearly or more than 60%. Especially in the brewing period, the proportion of reports with 0-5000 words reached 97%, while in the subsequent outbreak period, duration period, and recovery period, the proportion of reports with 0-5000 words decreased to about 60%, and the proportion of reports with more than 5000 words increased significantly, especially the amount of reports with 15000-20000 words increased rapidly from 0 in the brewing period to 106 in the outbreak period and 55 in the duration period. With the development of the COVID-19, the large-scale reports of “healthy China” have significantly increased, but the overall coverage remains small [24].

### 4.5. The Original Is the Core, and the Source of Contributions Will Be Expanded in the Middle and Later Stages

In terms of manuscript sources, the reports of “healthy China” in all stages are mainly original, and the original reports in the four stages account for more than 50%, reaching the highest in the recovery period, which is 65%. In addition, the amount of reports quoted from other mainstream media showed a gradual downward trend, with more than 40% in the gestation period and outbreak period, and fell to about 29% in the duration and recovery period. Through the analysis of the samples, it is found that the citations mainly come from the traditional mainstream authoritative media such as Xinhua news agency and people's daily and health news. In the first two stages of the severe epidemic situation, “healthy China” pays more attention to the quotation of information from the central media and party media, so as to ensure the authority and reliability of important information, answer audience doubts, and alleviate audience anxiety. In addition, the proportion of reports from social contributions and quoted from the media increased significantly during the duration, reaching 4.4% and 9.4%, respectively, and more attention was paid to the transmission of first-hand information from social groups, as shown in Table 8 [25].

### 4.6. Authoritative Departments Are the Primary Source of Information

As shown in Table 9, in terms of news sources, the main sources of “healthy China” reports at all stages are from national leaders and government officials, accounting for more than 50%. Among them, 73% of the reports in the gestation period are from national leaders and government officials, which decreased in the subsequent outbreak period and duration period, 59% and 56.2%, respectively, and rebounded to 65.8% in the recovery period. The proportion of reports with experts and scholars as the main source also decreased, from 16.2% in the gestation period to 11.1% and 3% in the outbreak period and duration period. On the other hand, the proportion of reports with medical staff as the main source has increased significantly, from 10.8% in the gestation period to 19.6% in the outbreak period, 24% in the duration period, and 20.7% in the recovery period, which are close to or more than twice the gestation period. The proportion of reports with people from all walks of life and the public as the main source has also increased from 0% in the gestation period to 4.4% and 7%. On the whole, during the epidemic, “healthy China” insisted on taking authoritative information from national leaders and government officials as the core source of its own reports and paid more attention to conveying the opinions and analysis of experts and scholars in the medical field during the gestation period when it was still unknown about novel coronavirus. As the epidemic gradually entered the outbreak period and duration, medical teams all over the country have supported all parts of Hubei, including B. Medical personnel have become the main force in the fight against the epidemic, and “healthy China” has also paid more attention to the report of information from medical personnel. At the same time, in addition to medical staff, a series of antiepidemic activities from all walks of life are also gradually spreading out during the outbreak and duration, and information from the police, grass-roots cadres, takeaway brothers, taxi drivers, and other people in all sectors of society and the public has also increased.

### 4.7. The Change Trend of Relevant Reports of the Government and the Medical System Is Opposite

The report topic is the most important category among all categories, which directly presents the core content reported by the three categories of WeChat official account. Government meetings, measures, and instructions were the main topics of coverage during the gestation period, accounting for 45.9%, and then decreased to 33.7%, 15.6%, and 17.5%, respectively. The work situation and advanced case reports of medical and epidemic prevention staff increased significantly after the gestation period, accounting for 21.3%, 29.9%, and 27.4%. A typical example occurred on February 7, when died after ineffective rescue. The reported amount of antiepidemic activities from all walks of life reached a peak during the duration, accounting for 6.9%. The proportion of epidemic prevention science popularization and troubleshooting reports was higher at the beginning of the epidemic, accounting for 27%, and then gradually fell, falling to 11.3% in the duration. The relevant reports on the production and living conditions of citizens during the epidemic period reached a peak in the duration, accounting for 13.1%. The resumption of work and production has been carried out in succession, and major cities across the country have gradually returned to normal production and living conditions. “Healthy China” has also paid more attention to the reports on this content. In addition, reports on the epidemic situation and prevention and control progress in various parts of the country, including Wuhan, peaked during the recovery period, accounting for 20.1%. Through the analysis of the samples, it is found that due to the overall control of the epidemic, the reports on government instructions and expert popular science content have been reduced, but at this time, all parts of the country still maintain a tight prevention and control situation, and the epidemic data notification in all regions of the country is still maintaining a certain frequency, so the proportion of such reports has increased in the recovery period. See Table 10 for details.

## 5. Analysis of Translation and Expression Strategies of Professional Terms in Publicity Reports of Public Emergencies

### 5.1. Strengthen Discourse Awareness and Establish a Holistic View

Due to the lack of textual awareness, there are a lot of cohesion problems. Most of these cohesion problems are caused by not thinking based on the text. Some studies believe that cohesion is a semantic concept, which refers to the relationship between the components in a text. Therefore, we can find that cohesive devices are not used groundlessly but serve the discourse. If the cohesive devices are used improperly, it will destroy the relationship between the textual components and make the text incoherent. Therefore, to choose appropriate cohesive devices, we must first establish discourse awareness, first understand the meaning of the whole text, and then choose cohesive devices.

### 5.2. Flexible Use of Cohesive Means

In addition to the rational use of these two strategies in publicity texts, another major feature is the use of a large number of cohesive devices. The rational use of cohesive devices can make the translation more coherent, and coherence is one of the important conditions for accurately conveying the information of the translation. The commonly used cohesive devices in publicity texts include reference, substitution, ellipsis, connection, and lexical means. Due to the formality of style, publicity texts have a high standard for the logic and coherence of language, and cohesive devices are one of the important means to achieve this standard.

There are great differences in cohesive devices between English and Chinese texts, because Chinese is a language that emphasizes “parataxis,” while English is a language that emphasizes “hypotaxis.” In Chinese expression, repetition is common and can be seen everywhere. However, in English, repetition should be avoided as much as possible, and some means, such as pronouns and synonyms, will be used to replace the expression that needs to be repeated. In terms of reference, there is little difference between English and Chinese. However, personal pronouns and demonstrative pronouns are used more frequently in English than in Chinese. In terms of substitution, English uses substitution more than Chinese, because Chinese is more inclined to reproduce the original word. In terms of ellipsis, because Chinese emphasizes “parataxis,” Chinese expression will not focus on form. English emphasizes “hypotaxis” and “ellipsis is accompanied by formal or morphological markers in many cases” In short, it is not that a textual cohesive device will only be used in Chinese, not in English, and vice versa. In other words, reference, substitution, ellipsis, and connection are used in both Chinese and English, but the frequency of use is different, and the difference in frequency stems from the different emphasis of the two languages.

As Chinese is our mother tongue, it deeply affects our way of thinking. In the process of translation, we are easily drawn by the original text and easily copy the cohesive devices of the original text, such as the interpretation of the conjunction “Huan” in example 7. In Chinese, “Huan” can refer to both simultaneous events and successive events. If it is directly corresponding to “also” in English, it is easy to cause the problem of unknown event time. Therefore, in the process of translation, we should be aware of the differences in cohesive devices between English and Chinese texts. We should not directly apply the cohesive devices in the Chinese original text into the translation but deeply analyze the logical relationship between words and sentences and reselect the appropriate cohesive devices.

### 5.3. Avoiding the Influence of Chinese Negative Transfer

Because we are deeply and long influenced by our mother tongue, we will always be influenced by our mother tongue Chinese in the process of second language acquisition. As English is our second language, it is difficult for us to reach the level of native speakers at present, and every translation project is an opportunity for us to exercise and learn, so we will inevitably be affected by Chinese in the process of translation. For example, in terms of lexical cohesion, it is difficult to make good use of “cooccurrence.” We often think of Chinese idiomatic collocations and then translate them into English. However, in English, such collocations are inappropriate, such as example 12. Therefore, when translating, we translators must be aware of the differences between Chinese and English languages, be able to jump out of the mother tongue circle, translate the text from the perspective of English readers, and strengthen our English thinking. Of course, to improve the use of cohesive devices, a lot of practice is essential. At the same time, we should also learn a lot of authentic English expressions and accumulate parallel texts to improve our level.

## 6. Conclusion

With the further deepening of globalization and the gradual improvement of China's international status, the demand for publicity translation is increasing. Publicity translation is aimed at introducing China to the outside world, covering politics, economy, culture, diplomacy, military, and many other aspects. It is one of the important ways for the world to understand China. As translators, we must be careful when doing publicity translation and use cohesive devices reasonably to make the translation coherent and logical, so as to accurately express the meaning of the text.

As a publicity text, in order to improve the translation level and the ability to use cohesive devices, the author collected and studied the problems related to textual cohesion encountered in the process of preliminary translation and divided them into two categories: grammatical cohesion and lexical cohesion. Then, carry out secondary classification, divide the grammatical cohesion problems into four categories (reference, substitution, ellipsis, and connection), and divide the lexical cohesion problems into two categories (repetition and lexical collocation (cooccurrence)). In each subcategory, we find some typical cases, dig deep into the meaning of the original text, analyze the initial translation problems, break through them one by one, and summarize the laws.

Language carries the history and culture of a nation, and translation is a bridge to help us cross the language gap. Therefore, translation plays an extremely important role in cultural exchange. A good translation must be able to accurately convey the meaning of the original text. In order to accurately express the meaning of the text, the translation must be coherent, and to achieve coherence, it must be supported by appropriate cohesive means. Cohesion is not a simple stacking of discourse components, but an analysis of the meaning of each component and the relationship between their components. Then, choose appropriate cohesive devices to reflect this relationship. Due to the limited research on translation and the lack of translation experience, this paper will inevitably have some deficiencies, but I hope this paper can provide some inspiration and reference for the translation of other publicity texts in the selection of cohesive devices.

## Figures and Tables

**Figure 1:** The process of translating manuscripts by translation companies (high-end).

**Figure 2:** News trend chart.

**Figure 3:** Strip chart of the report page of Southern Metropolis Daily.

**Figure 4:** Strip chart of the reporting genre of Southern Metropolis Daily.

**Figure 5:** Distribution map of topics reported by Southern Metropolis Daily.

**Figure 6:** Columnar distribution of sources of Southern Metropolis Daily.

**Figure 7:** Distribution of protagonists reported by Southern Metropolis Daily.

**Figure 8:** Distribution of reporting positions of Southern Metropolis Daily.

**Figure 9:** Report volume of “healthy China” at each stage.

**Figure 10:** Push time of “healthy China” at each stage.

**Figure 11:** Content presentation of “healthy China” at each stage.

**Figure 12:** Text length of “healthy China” at each stage.

**Table 1:** List of news framework research categories.

Category	Definition	Category formulation purpose	Theoretical basis for category formulation	Research questions
Report genre category	Expression form of report content	Different reporting genres have different functions, and choosing the appropriate reporting genres is conducive to achieve the communication effect.	Properly grasp and use the genre of news reports, and make news materials suitable for their place, without wasting materials.	What are the most used reporting genres in different types of media

Topic framework category	The core idea of news content	Understand that there are several news frames contained in the “poison capsule” event; positioning how different media frame the “poison capsule” event.	“News framework is the heart or main point of news content.”	What are the main theme frameworks presented, and how are the reporting frameworks of different types of media “poison capsule” events different

Source category	General provider or providing organization of newsletters	In the “poison capsule incident” report, which sources did the three media choose, and whether there was a bias in the choice of sources.	“The news sources are the competitors of social action, competing for the initiative of speaking and discourse in the media field. These competitors mobilize resources and manpower through the organizational culture, construct the speaking content in line with the organizational framework, and try to approach the media, so as to win their acceptance of the argument, become the core and basic position of the news framework, so as to affect the public and build the mainstream trend of thought in the society.”	What are the differences between different media in the choice of news sources, and the relationship between news sources and the formation of the framework

Report protagonist category	Key reporting objects in the news	Summarize what aspects of the “poison capsule incident” were highlighted by the three media.	Zhong Xiaowen: “the focus of every news report is to outline the essentials' it can be said that it is the theme embodiment of a news content.”	What are the main reporting objects, and how are the reporting objects of different media different

Report position category	Is the attitude of the report positive, negative or neutral	Grasping the reporting position will directly affect the scientific disposal of public health emergencies.	Modigliani: “only with active supporters can an issue achieve social reality.”	What is the reporting position? Are the reporting positions of different media the same

**Table 2:** Layout of the report of Southern Metropolis Daily.

Page	Southern Metropolis Daily	
	Number of reports	Proportion
Front page	4	6.0%
Front page of a newspaper	27	40.9%
Comment edition	10	15.1%
Domestic version	2	3.0%
International edition	0	0.0%
Economic edition	7	10.0%
Local news	12	19.0%
Urban edition	4	6.0%

**Table 3:** Distribution of report genres of Southern Metropolis Daily.

Reporting genre	Southern Metropolis Daily	
	Number of reports	Proportion
News	37	56.3%
Communication	10	15.2%
Exclusive interview	2	3.0%
Comment	12	18.0%
Popular science abstracts	4	6.0%
Other	1	1.5%

**Table 4:** Distribution of topics reported by Southern Metropolis Daily.

Report theme	Southern Metropolis Daily	
	Number of reports	Proportion
Incident investigation	16	24.0%
Case report	1	1.5%
Quality inspection and problem capsule treatment	20	30.3%
Government measures and disposal of relevant responsible persons	15	23.0%
Celebrity endorsement	3	4.5%
Other	11	16.7%

**Table 5:** Distribution of sources of Southern Metropolis Daily.

Source	Southern Metropolis Daily	
	Number of reports	Proportion
Government departments and officials	32	48.5%
Experts and scholars	7	10.6%
Enterprise group and person in charge	4	6.0%
Media and journalists	19	28.8%
Consumer	1	1.5%
Other	3	4.6%

**Table 6:** Distribution of protagonists reported by Southern Metropolis Daily.

Report protagonist	Southern Metropolis Daily	
	Number of reports	Proportion
Government departments and officials	22	33.3%
Enterprise group and person in charge	21	32.0%
Consumer	2	3.0%
Social groups or organizations	1	1.5%
Policies and regulations	5	7.6%
Drug safety knowledge	9	13.6%
Star	2	3.0%
Other	4	6.0%

**Table 7:** Distribution of reporting positions of Southern Metropolis Daily.

Reporting position	Southern Metropolis Daily	
	Number of reports	Proportion
Positive	5	7.6%
Neutral	49	74.2%
Negative	12	18.2%

**Table 8:** Manuscript sources of “healthy China” at each stage.

Manuscript source	Incubation		Outbreak period		Duration		Convalescence	
	Quantity	Proportion	Quantity	Proportion	Quantity	Proportion	Quantity	Proportion
Original	20	54%	437	54.6%	246	56.5%	346	65.0%
Quote other mainstream media	17	46%	322	40.3%	129	29.6%	152	28.6%
Quoted from media	0	0%	14	1.7%	19	4.4%	12	2.3%
Social contribution	0	0%	26	3.3%	41	9.4%	21	4.0%
Foreign media	0	0%	1	0.1%	0	0%	1	0.2%

**Table 9:** Sources of manuscripts at various stages of “healthy China.”

Source	Incubation		Outbreak period		Duration		Convalescence	
	Quantity	Proportion	Quantity	Proportion	Quantity	Proportion	Quantity	Proportion
National leaders and government officials	27	73.0%	473	59.0%	244	56.2%	350	65.8%
Experts and scholars	6	16.2%	89	11.1%	13	3.0%	20	3.7%
Medical staff	4	10.8%	157	19.6%	104	24.0%	110	20.7%
Patient	0	0%	5	0.6%	2	0.5%	1	0.2%
Foreign governments and international organizations	0	0%	15	1.8%	2	0.5%	1	0.2%
People from all walks of life	0	0%	35	4.4%	30	7.0%	5	1.0%
Other	0	0%	27	3.4%	39	9.0%	45	8.4%

**Table 10:** Topics reported at various stages of “healthy China.”

Report theme	Incubation		Outbreak period		Duration		Convalescence	
	Quantity	Proportion	Quantity	Proportion	Quantity	Proportion	Quantity	Proportion
Government meetings, measures, and instructions	17	45.9%	270	33.7%	68	15.6%	93	17.5%
Working conditions and advanced cases of medical and epidemic prevention staff	6	16.2%	171	21.3%	130	29.9%	146	27.4%
Treatment and living conditions of affected patients and suspected infected persons	0	0%	21	2.6%	6	1.4%	14	2.6%
Antiepidemic activities of all sectors of society	0	0%	25	3.1%	30	6.9%	23	4.3%
Epidemic situation and prevention and control progress in China, including B	4	10.8%	57	7.1%	55	12.7%	110	20.1%
Epidemic prevention and control in the world and other countries, and exchanges and cooperation between China and other countries	0	0%	12	1.5%	16	3.7%	10	1.9%
Epidemic prevention science popularization, explanation of doubts	10	27%	168	20.9%	49	11.3%	53	10%
Activities and conferences of the World Health Organization, the United Nations, and other international organizations, and exchanges and cooperation between China and international organizations	0	0%	19	2.4%	2	0.4%	7	1.3%
Various adverse phenomena occurred during the epidemic	0	0%	1	0.1%	6	1.4%	1	0.2%
Spiritual inspiration to people	0	0%	13	1.6%	12	2.8%	12	2.3%
Production and living conditions of citizens during the epidemic period	0	0%	43	5.4%	57	13.1%	54	10.1%
Other	0	0%	0	0%	4	0.1%	9	1.7%

## Data Availability

No data were used to support this study.

## References

[1] Xu C., Li Q. (2021). Machine translation and computer aided English translation. *Journal of Physics: Conference Series*.

[2] Bylina E. E., Skopintseva T. A., Sludneva L. V., Yurkovskaya E. A. (2020). Current trends in the development of logistics professional discourse terminology. *IOP Conference Series: Materials Science and Engineering*.

[3] Shen L. (2022). On translation of psychological terminology. *Open Journal of Social Sciences*.

[4] Xie X., Wu X., Wei X., Che C. (2021). A method of terminology alignment in historical books based on the correspondence between pivot language and position. *Journal of Physics: Conference Series*.

[5] Chen W., Cui K. (2022). Polymer crystallization under external flow. *Reports on Progress in Physics*.

[6] Ramesmayer C., Mitterberger M., Oberhammer L., Kunit T., Lusuardi L. (2021). Lower ureteral compression through external vascular elongation in a cyclist: a case report. *International Journal of Surgery Case Reports*.

[7] Narayanan V., Patel A., Mbogo J. (2022). Linear accelerator based external beam radiotherapy in glomus jugulare tumour: a retrospective review from a tertiary cancer hospital in Kenya. *Case Reports in Clinical Medicine*.

[8] Rajanna R. R., Natarajan S., Prakash V., Vittala P. R., Sahoo S. (2021). External cardiac loop recorders: functionalities, diagnostic efficacy, challenges and opportunities. *IEEE Reviews in Biomedical Engineering*.

[9] Wettstein A., Diddens D., Heuer A. (2021). Polymer electrolytes in strong external electric fields: modification of structure and dynamics. *Macromolecules*.

[10] Palmeri N., Locke A., Tung P. (2022). External defibrillation resulting in loss of ventricular capture during atrial lead testing. *Heart Rhythm Case Reports*.

[11] Hisanaga M., Nosanaka T., Maruta H., Maruyama K., Yamaguchi H. (2021). Transanal approach after preoperative imatinib treatment of a rectal gastrointestinal stromal tumors with external anal sphincter invasion: a case report. *International Journal of Surgery Case Reports*.

[12] Crossley E., Touska P., Thavaraj S., Connor S., Pai I. (2021). An unusual clinico-radiological presentation of epithelioid haemangioma as an external ear mass. *Otolaryngology Case Reports*.

[13] Poynard T., Lacombe J. M., Deckmyn O., Peta V., Carrat F. (2021). External validation of LCR1-LCR2, a multivariable HCC risk calculator, in patients with chronic HCV. *JHEP Reports*.

[14] Teh R. A., Hoshal S., Hoshal G. L. (2020). Bilateral external auditory canal masses following repair of ruptured abdominal aortic aneurysm and open decompressive exploratory laparotomy for compartment syndrome: a rare case of spontaneous bilateral otorrhagia. *Radiology Case Reports*.

[15] Ian G. (2020). A comparison of a moderately hypofractionated IMRT planning technique used in a randomised UK external beam radiotherapy trial with an in-house technique for localised prostate cancer. *Reports of Practical Oncology & Radiotherapy*.

[16] Zhang Y., Ascaso C., Martínez A. H., Sanchez J., Rovirosa A. (2020). Postoperative endometrial carcinoma treated with external beam irradiation plus vaginal-cuff brachytherapy. Is there a dose relationship with G2 vaginal complications?. *Reports of Practical Oncology and Radiotherapy*.

[17] Lee B. H. (2020). Anomalous external carotid-internal carotid artery anastomosis diagnosed by computed tomography angiography: a case report. *Radiology Case Reports*.

[18] Mukherjee A., Sharma N., Chakraborty M., Saha P. K. (2022). A study on the influence of external magnetic field on nitrogen RF discharge using Langmuir probe and OES methods. *Physica Scripta*.

[19] Mühlenpfordt I., Stritter W., Bertram M., Ben-Arye E., Seifert G. (2020). The power of touch: external applications from whole medical systems in the care of cancer patients (literature review). *Supportive Care in Cancer*.

[20] Tang L., Yishake M., Ye C., Hade H., Li Z., He R. (2020). Safe zone for lateral pin placement for external fixation of the distal humerus. *Clinical Anatomy*.

[21] Sharma A., Kumar R. (2019). Risk-energy aware service level agreement assessment for computing quickest path in computer networks. *International Journal of Reliability and Safety*.

[22] Ajay P., Nagaraj B., Pillai B. M., Suthakorn J., Bradha M. (2022). Intelligent ecofriendly transport management system based on IoT in urban areas. *Environment Development and Sustainability*.

[23] Chen J., Liu J., Liu X., Xu X., Zhong F. (2021). Decomposition of toluene with a combined plasma photolysis (CPP) reactor: influence of UV irradiation and byproduct analysis. *Plasma Chemistry and Plasma Processing*.

[24] Huang R., Zhang S., Zhang W., Yang X. (2021). Progress of zinc oxide-based nanocomposites in the textile industry. *IET Collaborative Intelligent Manufacturing*.

[25] Liu Q., Zhang W., Bhatt M., Kumar A. (2021). Seismic nonlinear vibration control algorithm for high-rise buildings. *Nonlinear Engineering*.

